The article "Diagnosis of Alzheimer's Disease Severity with fMRI Images Using Robust Multitask Feature Extraction Method and Convolutional Neural Network (CNN)" was published in 2021. Journal: Comput Math Methods Med.

# Diagnosis of Alzheimer's Disease Severity with fMRI Images Using Robust Multitask Feature Extraction Method and Convolutional Neural Network (CNN)

**DOI:** 10.1155/2021/5514839

**Published:** 2021-04-28

**Authors:** Morteza Amini, Mir Mohsen Pedram, AliReza Moradi, Mahshad Ouchani

**Affiliations:** ^1^Department of Cognitive Modeling, Institute for Cognitive Science Studies, Shahid Beheshti University, Tehran, Iran; ^2^Department of Electrical and Computer Engineering, Faculty of Engineering, Kharazmi University, Tehran, Iran; ^3^Department of Cognitive Modeling, Institute for Cognitive Science Studies, Tehran, Iran; ^4^Department of Clinical Psychology, Faculty of Psychology and Educational Science, Kharazmi University, Tehran, Iran; ^5^Department of Cognitive Psychology, Institute for Cognitive Science Studies, Tehran, Iran; ^6^Institute for Cognitive and Brain Science, Shahid Beheshti University, Tehran, Iran

## Abstract

The automatic diagnosis of Alzheimer's disease plays an important role in human health, especially in its early stage. Because it is a neurodegenerative condition, Alzheimer's disease seems to have a long incubation period. Therefore, it is essential to analyze Alzheimer's symptoms at different stages. In this paper, the classification is done with several methods of machine learning consisting of *K*-nearest neighbor (KNN), support vector machine (SVM), decision tree (DT), linear discrimination analysis (LDA), and random forest (RF). Moreover, novel convolutional neural network (CNN) architecture is presented to diagnose Alzheimer's severity. The relationship between Alzheimer's patients' functional magnetic resonance imaging (fMRI) images and their scores on the MMSE is investigated to achieve the aim. The feature extraction is performed based on the robust multitask feature learning algorithm. The severity is also calculated based on the Mini-Mental State Examination score, including low, mild, moderate, and severe categories. Results show that the accuracy of the KNN, SVM, DT, LDA, RF, and presented CNN method is 77.5%, 85.8%, 91.7%, 79.5%, 85.1%, and 96.7%, respectively. Moreover, for the presented CNN architecture, the sensitivity of low, mild, moderate, and severe status of Alzheimer patients is 98.1%, 95.2%,89.0%, and 87.5%, respectively. Based on the findings, the presented CNN architecture classifier outperforms other methods and can diagnose the severity and stages of Alzheimer's disease with maximum accuracy.

## 1. Introduction

In fluorodeoxyglucose-positron emission tomography research, cognitive impairment in AD has been correlated with localized brain metabolic damage in systematic and functional imaging experiments [1–3]. Blood-oxygen-level-dependent imaging was seen to reflect healthy functional networks, including default mode (DMN), visual (VIS), and executive networks (EN) [4], within a given resting state. Unlike task-related functional MRI (fMRI), patients' capability to recognize and memorize the instructions for executing a given task is not confounded by resting-state fMRI, which makes it useful for the survey of individuals with cognitive decline [5]. Besides, convincing literature-wide data confirms the application of resting-state connectivity as an AD biomarker [6]. Machine learning (ML) is an artificial intelligence field that typically utilizes factual methods to allow computers to “learn” through data from stored datasets. A subset of ML [7] is fundamental deep learning (DL). The DL is a neural network that uses several variables and layers to define. There are a variety of simple network architectures [8], including CNNs, mainly a standard spatial mutual weight neural network [9].

The CNN is designed to identify images that see the edges of a known target on the image by making convolutions inside [10]. (ii) Recurrent neural networks are names of artificial neural networks where a graph is generated by specific associations between nodes in the temporal chain. RNNs can use their internal condition to handle the sequences of inputs, unlike feedforward neural networks. RNN is meant to identify sequences such as a voice signal or a text [9], for example. (iii) In recursive neural networks, the input sequence does not include a time dimension, and the input must be hierarchically evaluated in a tree form [8, 10]. Various external inputs usually contribute to distinct brain functions, and various functional brain representations are displayed by different brain activities [11]. For that function, the classification of images plays an essential role in detecting various brain functions. Several deep learning approaches have recently been suggested to carry out image recognition for various brain activities [12, 13]. A deep neural network feedforward has been employed by Koyamada et al. [12] to identify different brain functions, including preferences; motor, social, emotional, and language activities; and work memory, using functional magnetic resonance imaging (fMRI) images. A SoftMax layer and various secret layers were used in the feedforward deep neural network. Similarly, to get high-level latent properties, these hidden layers were used. In contrast, the SoftMax layer has been applied to calculate a subject's ability in a class. To boost the final classification efficiency, dropout, minibatch stochastic decrease [14], and main sensitivity analyses [15] were also integrated into the deep feedforward neural network. Jang et al. newly exploited deep neural networks and hidden layers completely connected to feedforward to distinguish different sensor roles, including visual attention and stimuli and right-hand and left-hand clenching, are included. The DL classification of MRI images included other classifications above and below the classifications, such as diagnosis of stroke [16], age predictions [17], classification of attention-deficit hyperactivity disorder (ADHD) [18], prejudice against cerebellar ataxia [19], and predictive emotional response [20]. Due to science, computer-aided diagnosis systems (CADs) were developed to play an important role in enhancing the understanding of medical imagery among researchers and physicians. The application of the machine learning technique, in particular DL strategies in CAD models to diagnose and classify stable control patients with average (CN), AD, and mild cognitive impairment (MCI), has exponentially grown [21, 22]. The automatic diagnosis of AD performs an essential role in human health, especially in the early stages. AD has a considerable incubation period because it is a neurodegenerative disorder.

Thus, the AD symptoms need to be analyzed at various levels. Currently, several scholars have discussed using image classification to carry out AD diagnosis. Several DL approaches have been suggested to use MRI images to introduce multiple AD patients' severity [22, 23]. The higher the image quality, the better the outcomes achieved, known in image analysis. However, the quality of image relies on image processing, and when the picture is acquired higher, the image quality is higher. MRI retains noninvasive and good contrasting properties of soft tissue but does not expose to people ionizing with high radiation. As MRI can produce a great deal of priceless knowledge of tissue frameworks such as position, size, and type, more attention is paid to computerized diagnostics and clinical routine [24, 25]. Functional and structural imaging can be classified into MRI. T1-weighted MRI (T1w), diffusion tensor imaging (DTI), and T2-weighted MRI (T2w) [26] are used in structural imaging. Functional imagery includes functional MRI task status (ts-fMRI) and functional MRI resting state (rs-fMRI). Medical diagnostic data systems are employed for medical centers and doctors to treat diseases, and analytical tools to improve management and diagnosis are critical. Given the crucial function of medical data in humans' lives, computer scientists have been involved in this area. Healthcare professionals may make their decisions, including medical diagnoses and the effects of severe conditions, by contributing to the medical details' classification. In addition to the number of these conditions, a data collection of diseases comprises patient symptoms as characteristics. The extensive patient evidence available can be used for health treatment. Data mining may be used in medical center studies to provide appropriate origins of disease for prohibiting and prompt diagnosis and avoiding the significant costs of diagnostic tests [27].

In this paper, machine learning methods are utilized for Alzheimer's disease classification. Moreover, robust multitask methods are utilized for feature extraction of fMRI images from the ADNI dataset. In the output layer, the main aim is to find the severity of Alzheimer's diseases. Therefore, the results of MMSE are used. For classification and diagnosis of Alzheimer's disease severity, the machine learning methods are trained. Input and output features are applied for six classifiers including, KNN, SVM, DT, LDA, RF, and CNN. Finally, performance analysis consists of the confusion matrix and the ROC curve illustrates the classification results.

## 2. Research Background

AD recognition has been extended to many different methods focused on deep learning. Nevertheless, several controversial findings encouraged us to participate in the literature review to determine the current operating condition and what could be the potential innovations. In this section, the primary study concern is if DL techniques have been able to classify AD using neuroimaging data. The training dataset scale is considered to significantly impact the classifier's output over an undefined test range [28]. In each dataset, the amount of AD and MCI topics can be minimal, inadequate for deep models to be evaluated. For multimodality experiments, the condition is worse. Any experiments, however, have mixed datasets. While it can result in more heterogeneity by integrating multiple datasets, this may advance a broad and stable classification and prediction model. Using data augmentation is another means of addressing the small number of topics in a dataset. Data increase is a technique that increments the data range of training model applications without additional data being obtained. In approximately 20 percent of research aimed at enhancing classification performance, data enhancement strategies like random translation, rotation, reflection, adding noise, gamma filter, blurring, cutting, and scaling were used where appropriate [29].

Moreover, at various time points, longitudinal datasets include multiple brain scans per subject; it may also be employed for data increase in time, while their main objective was to analyze disease development [30]. While implementing a DNN from scratch is completed in some experiments, it is always impossible to do so: the training phase can use much time, or the sample may be tiny [31]. Even though there are millions of images in datasets of object detection and etiquette, neuroimaging datasets contain hundreds of images that help overfit the planning. It is generally beneficial to start tested, previously trained CNN with one dataset and retrain them with just the fine-tuning of CNN on another dataset (transfer learning). It is feasible since more general characteristics in the lower CNN layers can profit certain classification activities that can be moved from one program domain to another. CNN classifier is one of the effective methods for classification for all brain diseases. Besides, finding the best way for classification impacts diagnosis accuracy and process time. Therefore, our presented method is justified computationally.

Transfer learning is also more comfortable with small projects and produces higher performance than planning from the beginning [53]. Payan and Montana proposed classifying AD stages, namely, MCI, AD, and standard control [54] (NC). The algorithms were designed to implement a 3D CNN to separate brain scans employing autoencoding systems and 2D CNN. For 3D CNN and 2D CNN versions, an accuracy of 89.47 percent and 85.53 percent was reached. Liu et al. have also achieved a classification accuracy of about 85.53 percent with the identical network structure for 2D CNNs [34]. A study for the classification of AD was done by Sarraf and Tofighi [36]. The research was focused on classifying AD patients using MRI and fMRI scans from normal control subjects. For binary classification, two network architectures have been implemented. LeNet-5 and GoogleNet were the foundations for these CNN-based architectures. It obtained an approximate accuracy of 99 percent with LeNet and 100 percent with GoogleNet utilizing fMRI data. An analysis of research that focuses on AD classification using deep learning techniques is given in Table 1. Structural MRI or PET scans have been used in many experiments that concentrate on characterizing a few stages of the disorder, i.e., AD, MCI, and CN. In multiclass AD diagnosis and grouping, a restricted number of researches have employed fMRI findings.

## 3. Methods and Materials

### 3.1. Quantum Matched-Filter Technique (QMFT)

Initially, a preprocessing step with a noise reduction would take place. In conjunction with the local threshold and the active contour, each image is displayed employing a two-dimensional pixel array, the value of which is an integer in the [0, 255] scale. In two stages, local thresholds initialize images. Then, the input noise picture is named the main image to which image noise reduction is implemented. This procedure is used explicitly by the quantum matched-filter technique (QMFT) as a local search operator to improve the initial images. In this article, the utilization of local thresholds and active contours was considered since it is faster computationally than other approaches in the literature. Thus, there will be a decomposed picture at the end of the first stage. Thresholding is performed on the thorough coefficients in the second step, and each of the decomposed pieces is randomly picked and submitted to a reconstruction process. It is possible to describe the restoration portion [55]:

- Gaussian Blur: a Gaussian filter is used to filter an image. The filter size is chosen unintentionally, between 3 × 3 pixels and 5 × 5 pixels
- Mean filter (averaging filter): the picture is filtered utilizing an average filter
- Intensity change: a randomly selected associated criterion in [0.7, 1.3] range is used to multiply all the image pixels
- Integrate light-intensive parts that conduct the QMFT in quantum and reverse processing

Then, it executes the following procedures:

- One-point row: random selection of a pixel row
- One-point column: it is similar to the preceding method, except that it is regarded instead of a row
- Point-to-point random: every pixel is incorrectly chosen until a new image is produced from decomposition
- Mark points in rows and columns of the picture as QMFT to diminish the bulk of the noise

If the range value [0.1] chosen in the QMFT is lower than the rate of local search, the current image will be passed to the local search operator after a review. Its pixel value sorts the entire picture until the decomposition is complete. The best aspect ratio of the picture is then known in the sequel as a quantum value. The signal can be split into multiple displaced or revamped characteristic displays located at the feature's extraction point in fMRI photos. For the study of an image in its elements, local thresholds and active contours may be used. After implementing QMFT alongside local and active contouring thresholds, it is feasible to execute image classification operations. In this case, it is possible to destroy the local threshold coefficients and the QMFT-based active contour to delete certain information. Local thresholds and active contours based on QMFT have a significant advantage when details are separated into an image. It is possible to employ active contour to isolate excellent image information. Simultaneously, extensive details can be identified by local thresholds, integrating fine and extensive details and linearly and diagonally reading all rows and columns. Quantum reaches QMFT, so noise in the fMRI image can be minimized. A light display can be used to create a QMFT display with local thresholds and active contours. The local and active QMFT contouring mechanism has two key features: the oscillation or wave presence function, as in the following equation [55]:

(1) $$\begin{array}{c} {\left.\int_{-\infty }^{0}\Psi \left(t\right)\right|}^{2}dt<\infty . \end{array}$$

The energy in Ψ(*t*) is confined to a short period as

(2) $$\begin{array}{c} \int_{-\infty }^{0}\Psi \left(t\right)dt=0. \end{array}$$

Generally, the suggested approach is estimated to decrease the noise in

(3) $$\begin{array}{c} \Omega \left(I\right)=\left(\underset{\Omega }{\sum }\sqrt{1+\beta^{2}{\left|\nabla I\right|}^{2}}\right)+\frac{\lambda }{2}{\left(I-I_{0}\right)}^{2}. \end{array}$$

Within Equation (3), the term (*I* − *I*_0_)^2^ guarantees the rated image and a certain degree of authenticity and consistency in the original image, where *I* denotes the rated picture and *I*_0_ corresponds to the noisy picture. The parameter ∇*I* is described as the number of times of variable change, *β* and *λ* are balancing variables, and *Ω* is the sum of the image's pixels. The purpose of reducing Equation (3) is to diminish the broad variety of images while retaining accuracy and validation. For both *β* and *λ*, balancing values are modified from 1 to the image size to decrease Equation (3) [55].

### 3.2. Robust Multitask Feature

This paper is aimed at simultaneously catching common characteristics among several similar tasks and detecting outer work using the robust multitask learning function algorithm (rMTFL). The rMTFL will estimate the correct assessment and the true underlying weights. Also, if the true underlying weights are over noise thresholds, rMTFL will achieve exact sparsity patterns. Also, rMTFL optimization can be easily solved, and rMTFL scales can be used to solve significant problems [56]. Presume that there are *m* learning tasks relevant to the {(*X*_1_, *y*_1_), ⋯, (*X*_*m*_, *y*_*m*_)}, training results, where *X*_*i*_ ∈ *R*^*d*×*n*_*i*_^ is the *i*th task data matrix with column as a sample; *y*_*i*_ ∈ *R*^*n*_*i*_^ is the *i*th task response (*y*_*i*_ has continuous regression values and discrete classification values); *d* is the dimensionality of the data; and *n*_*i*_ is the number of *i*th task samples. The data were normalized to satisfy *X*_*i*_'s (*j*, *k*)th input, which is referred to as *x*_*jk*_^(*i*)^ [56]:

(4) $$\begin{array}{c} \overset{n_{i}}{\underset{k=1}{\sum }}{\left(x_{jk}^{\left(i\right)}\right)}^{2}=1,\;j\in {\mathbb{N}}_{d}. \end{array}$$

The linear function of learning is

(5) $$\begin{array}{c} y_{ii}\approx f_{i}\left(x_{j}^{\left(i\right)}\right)={\left(x_{j}^{\left(i\right)}\right)}^{T}w_{i},\;i\in {\mathbb{N}}_{m},j\in {\mathbb{N}}_{n_{i}}. \end{array}$$

The sum of two elements, *P* and *Q*, for each task and for decomposing of the weight matrix *W* = [*w*_1_, ⋯, *w*_*m*_ ] ∈ *R*^*d*×*m*^. To manipulate relationships between tasks, various regularization conditions on *P* and *Q* are used. The rMTFL model, theoretically, is developed as

(6) $$\begin{array}{c} \underset{W,P,Q}{\min}\;\overset{m}{\underset{i=1}{\sum }}\frac{1}{mn_{i}}{\left|\left|X_{i}^{T}w_{i}-y_{i}\right|\right|}^{2}+\lambda_{1}{\left|\left|p\right|\right|}_{1,2}+\lambda_{2}{\left|\left|Q^{T}\right|\right|}_{1,2}\;\\ \text{s}.\text{t}.\;W=P+Q. \end{array}$$

When *P* reports the mutual functions between tasks and *Q* learns the second term's outer tasks, *λ*_1_ and *λ*_2_ are nonnegative parameters to handle these two terms [56].

### 3.3. Convolutional Neural Network

CNNs have been widely employed for DL and the most prominent classes of neural networks, mostly in extensive data such as images and videos. It is a multilayer neural network architecture caused by cortex neurobiology. It consists of convolutional layers and fully connected layers. Between these two layers, subsampling layers can exist. The best of DNNs is achieved, which are challenging to scale along with multidimensional input data associated locally well. Therefore, CNN can be automatically applied in databases where comparatively large numbers of nodes and parameters are trained (e.g., image processing) [57].

#### 3.3.1. Convolutional Layer

This is the essential building block of a CNN that determines the output of associated inputs in the field of reception. These kernels' findings translate into data height and width, calculate the point product between inputs and filter values, and then create a 2D filter map enabled. It helps the CNN quickly find the filters that enable when an input temporarily detects a specific type of function [57].

#### 3.3.2. Nonlinearity Layer

Nonlinear characteristics have a high degree of importance and curvature. This layer's primary purpose is to convert the input signal into the output signal, which is used as an input in the next layer. Sigmoid or logistical forms, Tanh, ReLU, PReLU, ELU, and more, are not linear.

#### 3.3.3. Pooling Layer

The CNN may be locally or globally sampled to link the neuron outputs to an established neuron on a single layer in the following layer. The critical task is to limit the number of parameters and equations within the model to reduce spatial depiction volume [57]. It not only speeds up calculations but also takes the issue of overfitting into account. The most popular method of pooling is max pooling.

#### 3.3.4. Fully Connected Layer

FC layers are deep NNs typical for the regression or classification of the activation to construct the predictions. A description of the multilayer perceptron (MLP) neural system is equivalent to the typical neural system. The entire relationship with each activation is formed in the antecedent layer. Activation can be determined by the matrix multiplication and a bias offset [57].

#### 3.3.5. Loss/Classification Layer

The loss layer defines how the training eliminates the disparity between the actual and projected marks, ensuring that the training phase of NN is directly guided by it. Various loss functions for different commands such as SoftMax and crossentropy may be used in DCNN. SoftMax losses are used to measure a solo class of *K* mutually exclusive classes. The SoftMax layer is used to calculate the likelihood, i.e., the total output values for 1. Furthermore, this layer is a responsive max-output layer type, such that irregularities are distinguishable and often scalable. Sigmoid crossentropy loss is used to foresee *K*-free probability values [58]. The sigmoid capability yields negligible probabilities, and lines can be used for grouping various groups alongside these probabilities. A problem with sigmoid is that the gradient disappeared after the saturation had been achieved. Euclidean failure is used to regress to fully appreciated names. The following is an overview of the neural network model's programs, database, results, and implementations.

## 4. Results and Discussion

In this paper, machine learning methods are utilized for Alzheimer's disease classification. First of all, the input image is filtered with the QMFT method to reduced input fMRI images. To imply the classifier in fMRI images, feature extraction should be done for both the input and output layers. Therefore, robust multitask methods are used for feature extraction of input layers. Then, for reducing the number of features, the PCA method is chosen. In the output layer, the main aim is to find the severity of Alzheimer's disease. Therefore, the results of MMSE are the best choice. It consists of four categories: the low, mild, moderate, and severe patients' severity. The next step is to train the machine learning methods. Input and output features are applied for six classifiers including, KNN, SVM, DT, LDA, RF, and CNN. Finally, performance analysis consists of the confusion matrix and the ROC curve illustrates the classification results. The conceptual diagram of the method is presented in Figure 1.

### 4.1. Preprocessing of Dataset

Data used in this paper's preparation was obtained from the ADNI database. Each subject's standard format was a series of 140 64 × 64 × 48 3D NIFTI files and a single T1-weighted structural MRI file. Each 3D NIFTI file represented the patient's brain's rs-fMRI data from a 3-Tesla MRI scanner. Multiple subjects had nonstandard fMRI size (e.g., 96 × 96 × 48, 80 × 80 × 48) and were filtered out as well.

First, subjects were arbitrarily categorized into groups for training and testing. Around 80 percent of the details were required for training, and the remaining 20 percent was used for testing. For the training and testing datasets, similar preprocessing was implemented. First, the skull and neck voxels, which are the MRI scans' nonbrain regions, were removed from the T1-weighted image that corresponded to each subject. The resting-state fMRI contained 140 time steps per subject and was corrected for motion artifacts. Then, regular slice timing correction was applied to each time series because later steps assume all slices were acquired halfway through the relevant acquisition time. Slice timing correction shifts each time series by the appropriate fraction. Spatial smoothing was carried out next using a Gaussian kernel (5 mm full width at half maximum). Then, low-level noise was removed from the data using quantum matched-filter technique (QMFT). The noise reduction results can be shown by the 2D section of images in Figure 2.

Based on the results of QMFT in Figure 2, the prominent image noise was removed from 3D fMRI images. For better illustration of noised and reduced images, the contour form of image matrixes is shown in Figures 2(b) and 2(d). The peak signal-to-noise ratio (PSNR) is shown in Figure 3. Results of reduction for 140 images are depicted in Figure 3. The average value of PSNR for the tested images is 83.9731. The reduction of noise gives an exciting outcome that enables a proper extraction of features.

### 4.2. Feature Extraction and Input Features

The ADNI database is adopted for feature extraction of fMRI images. The fMRI of 675 patients is included in the results. fMRI data include 285 features classified into five types: average cortical thickness, the standard deviation of cortical thickness, the volume of cortical parceling, white matter, and surface area. The result is the score from 6 separate time points of the Mini-Mental State Examination: M06, M12, M18, M24, M36, and M48. The samples that fail to track the consistency of fMRI and missing results are removed.

### 4.3. Mini-Mental State Exam (MMSE)

According to certain risk factors, the cognitive function can decrease (e.g., hypertension, elevated cholesterol, cardiac arrhythmias). The physical and life quality of older people may be adversely affected. Dementia is a significant disorder and a cause of elderly disabilities. The second leading source in the dementation of AD is brain vascular disease or multi-infarct dementia. The Mini-Mental State Exam (MMSE) is an elderly cognitive function test commonly used; it requires orientation, attention, memory, language, and visual-spatial ability. The MMS is broken into two parts; the first only includes vocal responses and encompasses orientation, memory, and attention; 21 is the highest score. The second section checks the ability to name, obey verbal and written orders, automatically write a phrase, and copy a complex Bender-Gestalt figure-like polygon; the highest score is 9. Patients with seriously affected vision can have some added difficulties due to the reading and writing involved in part II, which can typically be eased by broad writing and allowed for in the scoring. There is a full cumulative score of 30 [59] (see Table 2).

For this paper, the relationship between Alzheimer's patients' functional magnetic resonance imaging (fMRI) images and their MMSE scores is assessed. Furthermore, a machine learning model's training is done on sample data consisting of 285 features (extracted from an fMRI image) and the patients' respective MMSE scores. The training data contained information for 800 patients with normalized features. The test sample consists of 200 datasets of features and a corresponding MMSE score as well.

### 4.4. Dimensionality Reduction

For function collection and reduction, the well-known PCA approach is used. PCA is a commonly utilized strategy for reducing dimensionality, extraction of features, and visualization of results. PCA can be described as the information's orthogonal projection into a low-dimensional, linear space known as the principal spaces. The predicted data variance rises. PCA diminishes the mean projection cost, defined as the mean square distance between the data points and their projections [60]. The value of characteristics is sorted in a descending order to find a sufficient number of characteristics. The total standard value summation (NCSE(i)) is then calculated as the corresponding sorted value:

(7) $$\begin{array}{c} \text{NCSE}\left(i\right)=\frac{\sum_{n=1}^{i}\text{e}\text{igenvalue}\left(n\right)}{\sum_{n=1}^{N_{f}}\text{e}\text{igenvalue}\left(n\right)},\;1\leq i\leq N_{f}, \end{array}$$

where the *n*th function's value is eigenvalue (*n*) and the dimensionality of the function vector obtained by the PCA method is *N*_*f*_. The result of feature reduction is depicted in Figure 4. Based on the chart, the minimum value of features with maximum variance should be chosen. Based on results, 167 features contain 98% variance of all 285 features. Therefore, classification should continue with these 167 features, regarding this reduction number of features decremented by 41.4%.

The results of classification with several methods of machine learning consisting of KNN, SVM, decision tree (DT), linear discrimination analysis (LDA), and random forest (RF) are illustrated in Figure 5. Regarding the confusion matrix of Figure 5, the green arrays show the true values, and red elements indicate false ones. The classification is performed based on four classes, including low, mild, moderate, and, severe based on the MMSE scoring system. The horizontal gray cells indicate sensitivity, and vertical cells illustrate precision values for each class. For instance, in the SVM method, from 690 patients with low severity, 656 (94.1%) are diagnosed correctly. However, 30 of them are misdiagnosed with mild, and four are detected with moderate severity. In other words, the sensitivity of low, mild, moderate, and severe is 95.1%, 57.6%, 84.9%, and 100%, respectively. Moreover, in the RF classifier, from all detected patients in the mild class, 97.7% (precision) are true. On the other hand, the precision of low, mild, moderate, and severe classes for RF classifier is 82.5%, 97.7%, 100%, and 100%, respectively. The value of the lower-right corner cell in the confusion matrix is the total accuracy value. To conclude, the results show that the accuracy of KNN, SVM, DT, LDA, and RF methods is 77.5%, 85.8%, 91.7%, 79.5%, and 85.1%, respectively. Moreover, the total error value of the classifier is illustrated in the lower-right corner with red text. Results indicated that from all traditional classifiers, DT results with high accuracy than other methods.

For a better analysis of the machine learning classifiers, the ROC curve is represented in Figure 6. For each of the classes, the ROC curve is different because it is plotted based on binary classification. The horizontal axis displays the ROC curve's false-positive trend, and its vertical axis shows the true-positive rate. In other words, the ROC curve is depicted, with consideration of each class as the positive state. Based on the ROC curve, if the values are observed with a low, false-positive rate and high true-positive rate, it is considered desirable. One of the essential criteria for the classifier's performance analysis is the area under the curve of ROC curve called AUC. It can be seen that the DT classifier resulted in high AUC than other methods. Furthermore, the AUC value for the severe class is almost identical, almost 100%.

Based on robust multitask features and MMSE score results, a CNN architecture for assessing or diagnosing Alzheimer's patient severity in this article is presented. The input layer consists of 167 features for every 1000 patients. Therefore, input matrix size is 167 × 1. For the convolutional layer, 16 filters with 5 × 5 size are used with stride [1] and zero padding. Moreover, for activating the layers, the ReLU function is used to vanish the negative values. Then, four fully connected layers are used with 384, 384, 384, and 4, respectively. Finally, the SoftMax layer is used to find probability and to activate the final layers. Then, the classification layer is used based on the crossentropy considering mutually exclusive classes. The architecture of the CNN layer is shown in Table 3.

The results of the classification process are indicated in Figure 7. The process is performed with core i7, Intel processor with 3 GHz CPU and 12GB RAM. The training process is done for 420 iterations. The accuracy and loss value of the training process is depicted in Figure 7. Furthermore, the confusion matrix of the presented CNN method is illustrated in Figure 8. Based on the low, mild, moderate, and severe status of Alzheimer patients, the sensitivity is 98.1%, 95.2%, 89.0%, and 87.5%, respectively. Moreover, the precision value for low, mild, moderate, and severe is 98.1%, 92.4%, 97.0%, and 100%, respectively. The absolute accuracy is also 96.7%. The summary of the results and comparison of the different classifiers are indicated in Table 4.

The results of the comparison between the presented architecture and traditional machine learning methods are shown in Table 4. Based on results, the sensitivity of the presented method outperforms other approaches. The sensitivity indicates the power of the method to diagnose disease severity based on the inputs. Therefore, the magnitude of it represented the potential of the classifiers. In other words, the sensitivity of the proposed CNN architecture is higher than that of other methods. The precision also shows the potential of results or reliability of the method. For instance, the precision of the CNN method is 98.1% for the low class. It means that, from all patients that the CNN recognized as low-severity patients, 98.1% are correct. To conclude the results, the presented CNN method's accuracy is 96.7% and higher than other methods. In the next priority, DT, SVM, RF, LDA, and KNN indicate high accuracy, respectively.

## 5. Conclusion

AD is an incurable brain illness affecting a large percentage of the planet. To enhance patients' lives and establish effective care and targeted drugs, early detection of AD is critical. The machine learning approaches are used to diagnose the seriousness of AD focused on fMRI images. To start the training process, matched-filter technique is applied to increase the contrast of the 3D images and decrease the noise or outlier of images. The ADNI containing fMRI data of 675 patients is used. The fMRI data include 285 features base on the robust multitask feature learning algorithm. The response (target) is the Mini-Mental State Examination score that shows the severity of AD including low, mild, moderate, and severe categories.

Furthermore, the machine learning model's training task is implemented using sample data consisting of 285 features (extracted from an fMRI image) and the patients' respective MMSE scores. The training data contained information for 800 patients with normalized features. The test sample consists of 200 datasets of features and a corresponding MMSE score as well. Then, the PCA approach is used for feature selection and reduction. Based on results, 167 features contain 98% variance of all 285 features. The classification is performed with several machine learning methods consisting of KNN, SVM, DT, LDA, random forest (RF), and CNN. The results show that the accuracy of the KNN, SVM, DT, LDA RF, and presented CNN method is 77.5%, 85.8%, 91.7%, 79.5%, 85.1%, and 96.7%, respectively. For the presented CNN architecture, for the low, mild, moderate, and severe status of Alzheimer patients, the sensitivity is 98.1%, 95.2%,89.0%, and 87.5%, respectively. Moreover, the precision value for low, mild, moderate, and severe is 98.1%, 92.4%, 97.0%, and 100%, respectively. In the next priority, DT, SVM, RF, LDA, and KNN indicate high accuracy, respectively. The detection of the severity of AD could help discover medications by having improved pathogenesis for evaluating the efficacy of target therapies that can delay the development of the disease. It can help recognize patterns of brain structural changes associated with the progression of Alzheimer's by combining clinical imaging with DL methods that can help identify risk factors and prognostic markers.

## Figures and Tables

**Figure 1:** The conceptual flowchart of the presented process.

**Figure 2:** Results of noise reduction using QMFT: (a) input image; (b) input image contour form; (c) noise-reduced image; (d) contour form of noise-reduced image.

**Figure 3:** The PSNR value of noise reduction from fMRI images.

**Figure 4:** The cumulative summation of sorted eigenvalues.

**Figure 5:** Confusion matrix of machine learning methods.

**Figure 6:** ROC curves of machine learning methods.

**Figure 7:** The accuracy and the loss value for the presented CNN architecture.

**Figure 8:** The confusion matrix of the presented CNN method.

**Table 1:** Summary research on Alzheimer's disease diagnosis methods.

Author	Year	Database	Modality	Method	Accuracy
Suk and Shen [32]	2013	Alzheimer's Disease Neuroimaging Initiative (ADNI)	PET, MRI, CSF	Stacked autoencoder, SVM	95.9
Suk al.[33]	2014	ADNI	PET, MRI	Deep Boltzmann machine	95.4
Liu et al. [34]	2016	ADNI	MRI	Influence of subclass number, multiview feature extraction, subclass clustering-based feature selection, SVM	93.8
Zu et al. [35]	2016	ADNI	PET, MRI	Label-aligned multi-task feature selection, support vector machine	96.0
Sarraf and Tofighi [36]	2016	ADNI	fMRI	LeNet-5	96.85
Sarraf and Tofighi [37]	2016	ADNI	MRI, fMRI	LeNet, GoogleNet	98.84
Li et al. [38]	2017	ADNI	MRI	CNN	88.31
Amoroso et al. [39]	2018	ADNI	MRI	Random Forest, deep neural network, fuzzy logic	38.8
Liu et al. [40]	2018	ADNI	MRI, PET	2D and 3D CNN,	93.26
Yang et al. [41]	2018	ADNI	MRI	The convolutional neural network, 3DVGGNET, 3DRESNET	76.6
Wang et al. [42]	2018	Open Access Series of Imaging Studies	MRI	CNN	97.65
Khvostikov et al. [43]	2018	ADNI	MRI, DTI	CNN	96.7
Shi et al. [44]	2018	ADNI	MRI, PET	Multimodal stacked deep polynomial network, SVM	97.13
Ramzan et al. [45]	2019	ADNI	fMRI	Off-the-shelf and fine-tuned	97.88
Parmar et al. [46]	2020	ADNI	fMRI	3D CNN	96.55
Duc et al. [47]	2020	ADNI	fMRI	3D CNN and SVM-RFE	85.27
Li et al. [48]	2020	ADNI	4D fMRI	3D CNN and C3d-LSTM	89.47
Al-Khuzaie et al. [49]	2021	Alzheimer Network (AlzNet)	2D fMRI	CNN	99.30
Bhaskaran and Anandan [50]	2021	Research Anthology on Diagnosing and Treating Neurocognitive Disorders	rsfMRI	Graph metrics and lateralization	97.54
Luo et al. [51]	2021	Population-specific Chinese brain atlas	rsfMRI	Graph metrics and false discovery rate (FDR)	95.67
Ahmadi et al. [52]	2021	Harvard Medical School	MRI	Robust PCA and CNN method	96

**Table 2:** Scoring system of MMSE and the severity of Alzheimer's disease.

Score	Severity	Psychometric analysis	Day-to-day functioning
25-30	Low	If there are clinical symptoms of cognitive disability, a formal cognition test can be useful	Clinically significant, however mild, deficits may be available. Only the most stressful everyday life tasks are expected to be affected
20-25	Mild	To further assess the trend and nature of deficits, a systematic examination can be useful	Meaningful effects. Any monitoring, assistance, and aid may be needed
10-20	Moderate	The formal assessment of whether there are clear health indications may be helpful	Obvious deficiency. 24-hour surveillance could be required
0-10	Severe	The patient will not be testable	Impairment labelled. 24-hour surveillance and support with ADL are likely to be required

**Table 3:** The architecture of the presented CNN method.

Layer	Type	Properties
1	Feature input	167 × 1 × 1 images
2	Convolution	16 (5 × 5) convolutions with stride [1]
3	ReLU	*F*(*x*) = max(0, *x*)
4	Fully connected	384 fully connected layer
5	Fully connected	384 fully connected layer
6	Fully connected	Four fully connected layer
7	SoftMax	$\sigma {\left(x\right)}_{i}=\frac{e^{x_{i}}\;}{\sum_{j=1}^{K}e^{x_{j}}},\;i=1,\cdots ,K\;x=\left(x_{1},\cdots ,x_{K}\right)$
8	Classification output	For multiclass grouping problems with mutually exclusive groups, the crossentropy loss

**Table 4:** Comparison of the diagnosis methods used in this paper.

	Class	KNN	SVM	DT	LDA	RF	Presented CNN
Sensitivity	Low	94.6%	95.1%	94.9%	91.0%	99.9%	98.1%
	Mild	51.1%	57.6%	94.3%	50.2%	54.6%	95.2%
	Moderate	6.8%	84.9%	61.6%	61.6%	47.9%	89.0%
	Severe	0.0%	100%	12.5%	87.5%	25.0%	87.5%

Precision	Low	79.0%	86.5%	96.9%	83.4%	82.5%	98.1%
	Mild	70.1%	80.0%	80.6%	70.6%	97.7%	92.4%
	Moderate	83.3%	89.9%	83.3%	61.6%	100%	97.0%
	Severe	0%	100%	50.0%	63.6%	100%	100%

Accuracy		77.5%	85.8%	91.7%	79.5%	85.1%	96.7%

## Data Availability

Data used in this paper's preparation was obtained from the ADNI database (http://adni.loni.usc.edu/).
